RETRACTED

# Increased EHHADH Expression Predicting Poor Survival of Osteosarcoma by Integrating Weighted Gene Coexpression Network Analysis and Experimental Validation

**DOI:** 10.1155/2021/9917060

**Published:** 2021-05-03

**Authors:** Juncheng Cui, Guoliang Yi, Jinxin Li, Yangtao Li, Dongyang Qian

**Affiliations:** ^1^Department of Orthopedic Surgery, The First Affiliated Hospital of University of South China, 69 Chuanshan Road, Hengyang, Hunan 421001, China; ^2^Department of Orthopaedics, The First Affiliated Hospital, Guangzhou Medical University/Guangdong key Laboratory of Orthopaedic Technology and Implant Materials, Guangzhou 510120, China

## Abstract

Enoyl-CoA hydratase and 3-hydroxyacyl CoA dehydrogenase (EHHADH), a member of the 3-hydroxyacyl-CoA dehydrogenase family, were previously demonstrated to be involved in the tumorigenesis of various cancer types. This study is aimed at determining of the diagnostic and prognostic value of EHHADH in osteosarcoma (OS). The overexpression of EHHADH was found both in OS and also other sarcoma types, and according to the retrospective cohort study, the EHHADH level was related to the overall survival and disease-free survival of the OS patients. Furthermore, knockdown of EHHADH under the influence of EHHADH small interfering RNA significantly suppressed the proliferation ability of the tumor cells. Moreover, EHHADH overexpressed was found in human OS tissues. In summary, the progression of OS could be enhanced by EHHADH, which may be a potential diagnostic and prognostic biomarker for OS patients.

## 1. Introduction

Osteosarcoma (OS) is one of the commonly occurring malignant tumors in bone tissues [1]. OS is derived from the mesenchymal cell line, and the frequent growth of the tumor is associated with the development of tumor osteoid (either direct or indirect manner) and bone tissue through the cartilage stage [2]. OS can typically be characterized by the high proliferation of the tumor cells, rapid metastasis, and high mortality rate [3]. However, medical failure of OS is the main issue which in turn results in the poor curative effect for OS [4]. Despite the huge development of therapeutic strategies, only lesser advancement in the treatment of OS patients has been obtained [5]. Currently, there are very few feasible biomarkers present that are involved in the determination of tumor burden and assess the therapeutic response for OS [6]. Hence, the discovery of efficient biomarkers for early diagnosis and prognostic evaluation of OS is greatly required. Therefore, the survival of the patients can be improved because of the development of early therapy for OS.

Enoyl-CoA hydratase and 3-hydroxyacyl CoA dehydrogenase (EHHADH), a member of the 3- hydroxyacyl-CoA dehydrogenase family, previously been reported to be involved in tumorigenesis of various types of cancer [7, 8]. Various studies have reported that several tumor-related diseases are enriched with EHHADH, which is of great importance for the progression of cancers [9, 10]. Thus, it is reasonably assumed that EHHADH is involved in the development of tumor-related diseases. However, only a few reports are suggesting the diagnostic role of EHHADH in the development of OS.

RETRACTED

Therefore, this study initially pursued the investigation of the prognostic value of EHHADH in OS. The overexpression of EHHADH was observed in both OS and other sarcoma types. According to the retrospective cohort study, the EHHADH level was related to the disease-free survival and overall survival of the OS patients. Furthermore, the clinical importance of EHHADH level in human OS and the regulatory effect of EHHADH on OS cell proliferation were explored.

## 2. Materials and Methods

### 2.1. TCGA Analysis

We obtained the data sets of sarcoma patients from TCGA Data Portal (https://tcga-data.nci.nih.gov/tcga/). The DEGs analysis was performed with the edge*R* package and visualized using the pheatmap *R* package. The volcano result was visualized with the ggplot2 *R* package. Results were reported as the average expression value of repeated genes. A two-tailed test was carried out between the two groups. *p* < 0.05 and ∣logFC | >1 were considered as differentially expressed genes.

### 2.2. Enrichment Analysis for Gene Ontology (GO) and Kyoto Encyclopedia of Genes and Genomes (KEGG) Pathway

The online tool Database for Annotation, Visualization, and Integrated Discovery version (DAVID) Bioinformatics Resources 6.8 was used to recognize the biological meaning of the listed genes. Analyses for the enrichment of the KEGG pathway and GO were performed with DAVID. We selected the GO and KEGG terms with FDR < 0.05.

### 2.3. Construction of the Protein-Protein Interaction (PPI) Network and Identification of Hub Genes

With the help of the PPI network, further information was obtained regarding the functional interactions between the DEGs. DEGs were imported into Search Tool for the Retrieval of Interacting Genes (STRING, http://www.string-db.org), and interactions with a combined score of >0.9 were identified. After that, with the help of the Cytoscape software (version 3.7.2), a PPI network was built. With the plugin software cytoHubba, hub genes were identified by degree analysis. The interaction between GO terms was visualized with clueGO, a plugin software of Cytoscape.

### 2.4. Oncomine Analysis

Oncomine (http://www.oncomine.org) integrates RNA and DNA-seq data from GEO, TCGA, and published literature. We can use Oncomine for the analysis of the differentially expressed genes, clinical correlation, and multigene coexpression. The coexpressed genes of EHHADH in sarcoma were retrieved from Oncomine with the default setting of fold change > 2 and *p* value < 0.01.

RETRACTED

### 2.5. The Analysis of Kaplan-Meier Plotter Survival

DEG prognostic values and coexpressed genes of EHHADH in sarcoma were further assessed by the examination of overall survival using the Kaplan-Meier plotter (http://kmplot.com/analysis/). It is an online tool that is used to assess the role of 54,675 genes on the survival of 13,316 cancer samples in 21 cancer types. The database sources include the EGA, GEO, and TCGA. The main purpose of the tool is the discovery and validation of meta-analysis-based biomarkers. Statistically significant results were showed *p* < 0.01.

### 2.6. Cell Culture and Transfection

OS cell line MG63 was obtained from the Shanghai Cell Bank (Shanghai, China), and DMEM and 10% fetal bovine serum (Thermo Fisher Scientific, Waltham, MA, USA) were applied to the cell culture at 37°C in 5% CO_2_. For transfection, the negative control small interfering RNA (siRNA) and EHHADH siRNA were designed by Suzhou GenePharma Biotechnology Co., Ltd. (Suzhou, China). Transfection of MG63 cells was performed with 50 nM NC siRNA or EHHADH siRNA and Lipofectamine 3000 (Thermo Fisher Scientific, Waltham, MA, USA).

### 2.7. Quantitative Reverse Transcription Polymerase Chain Reaction (qRT-qPCR)

Invitrogen TRIzol (ThermoFisher, Waltham, MA, USA) was used for the extraction of the total RNA from the OS cells and tissues according to the instructions of the manufacturer. To assess the EHHADH mRNA level, the qRT-PCR analysis was applied using a One-Step RT-PCR kit (Beijing Suolaibao Bio, Inc., Beijing, China) according to the instruction provided by the manufacture. The CBX3 primers were designed by Suzhou GenePharma Co., Ltd. (Suzhou, China) and are as follows: EHHADH forward, 5′-ATGGCTGAGTATCTGAGGCTG-3′ and reverse, 5′-ACCGTATGGTCCAAACTAGCTT-3′; and GAPDH forward, 5′-ACTGCGAATGGCTCATTAAATCA-3′ and reverse, 5′-AGCTCTAGAATTACCACAGTTATCCAAGT-3′. Cyclin D1 forward, 5′-TTGCCCTCTGTGCCACAGAT-3′ and reverse, 5′-TCAGGTTCAGGCCTTGCACT-3′. Cyclin D3 forward, 5′-CTGGCCATGAACTACCTGGA-3′ and reverse, 5′-CCAGCAAATCATGTGCAATC-3′.The 2^-*ΔΔ*Cq^ approach was used to quantify the EHHADH mRNA level.

### 2.8. Western Blot (WB) Analysis

The BCA method (ThermoFisher, Waltham, MA, USA) was applied to assess the concentration of proteins. Subsequently, the separation of equal amounts of the total protein was performed by using 12.5% SDS-PAGE, and then we transferred the separated proteins onto polyvinylidene difluoride membranes. To block the membrane, 5% skim milk was used at room temperature for 2 hours and was subjected to incubation with anti-EHHADH (1 : 800 dilution) (cat. no. Ab136059, Abcam) antibody or anti-GAPDH (1: 2,500 dilution) (cat. no. ab9485, Abcam). GAPDH was used as the internal reference to normalize the expression EHHADH.

RETRACTED

### 2.9. Statistical Analysis

Data are depicted as means ± SD, and all the statistical analyses were conducted by using GraphPad Prism 8.0 (GraphPad Software, CA, USA). Data comparison was based on Student's *t*-tests and one-way ANOVAs with Tukey's posthoc test as appropriate. The significant threshold was mentioned as *p* < 0.05.

## 3. Results and Discussion

### 3.1. TCGA Analysis

Through the TCGA database, we obtained the mRNA expression and clinical information of 265 cases (263 sarcoma patients and 2 normal people). After normalization of the data and comprehensive analysis, 912 downregulated and 21 upregulated DEGs were identified (Figure 1).

### 3.2. GO and KEGG Pathway Enrichment Analysis of DEGs

The DEGs were significantly involved in the biological progress of the metabolic process, excretion, fatty acid beta-oxidation, transmembrane transport, sodium ion transport, and oxidation-reduction process; in cellular components of the extracellular exosome, apical plasma membrane, mitochondrial matrix, mitochondrion, brush border membrane, an integral component of the plasma membrane, basolateral plasma membrane, and peroxisomal matrix; in molecular functions of electron carrier activity (Figures 2(a) and 2(b), Table 1); and in KEGG pathways of metabolic pathways, biosynthesis of antibiotics pathway, degradation pathway of leucine valine, and isoleucine, metabolism pathways of carbon, glyoxylate and dicarboxylate, propanoate, and fatty acid degradation pathway, proximal tubule bicarbonate reclamation pathway, peroxisome pathway, pyruvate metabolism pathway, etc. (Figure 2(c), Table 2).

### 3.3. Construction of the PPI Network and Identification of Hub Genes

The construction of an interaction network of DEGs was accomplished in Cytoscape (Figure 3(a)). DEGs were ranked by degree value in Cytoscape (Figure 3(b)). The top ten genes were EHHADH, ACOX1, AGXT, HMGCL, PIPOX, SLC27A2, DLD, ACADM, CAT, and DAO. They are considered hub genes. EHHADH was ranked No. 1 with a lesser *p* value.

### 3.4. The Kaplan-Meier Plotter Survival Analysis of Hub Genes

EHHADH was found to be linked with a shorter overall survival rate among ten hub genes while longer overall survival was associated with PIPOX, ACOX1, and SLC27A2 (*p* < 0.05) (Figure 4).

RETRACTED

### 3.5. Oncomine Analysis

The coexpressed genes of EHHADH were identified using a coexpression online tool in Oncomine. Results of the analysis revealed that the top ten coexpressed genes with the smallest correlation factor include DMGDH, BHMT2, TMEM37, DAB2, TLR3, GAL3ST1, SLC5A10, SLC17A3, CHST13, and CID3B (Figure 5).

### 3.6. The Kaplan-Meier Plotter Survival Analysis of EHHADH-Coexpressed Genes

For the ten coexpressed genes of EHHADH in sarcoma, DMGDH, BHMT2, TMEM37, TLR3, SLC17A3, and CID3B were associated with longer overall survival (*p* < 0.05) (Figure 6).

### 3.7. GO and KEGG Pathway Enrichment Analysis of EHHADH-Coexpressed Genes

EHHADH-coexpressed genes were significantly involved in the biological progress of negative regulation of the following: glucuronosyltransferase activity, cellular glucuronidation, and fatty acid metabolic process; in cellular components of the extracellular exosome, apical plasma membrane, and integral plasma membrane components; in molecular functions of retinoic acid binding, glucuronosyltransferase activity, transferring hexosyl groups, and transferase activity (Figures 7(a) and 7(b)); and in KEGG pathways of drug metabolism—other enzyme pathway, drug metabolism—cytochrome P450 pathway, metabolism of xenobiotics by cytochrome P450 pathway, etc. (Figure 7(c), Table 3).

### 3.8. Inhibition of EHHADH Suppresses MG63 Cell Proliferation

To detect the EHHADH expression in the OS tissue, qRT-PCR analysis was used to compare the EHHADH level between OS tissue and the adjunct bone tissue, and as shown in Figure 8(a), significantly increased level of EHHADH mRNA was found in the OS tissues compared with adjacent bone tissues. Next, to explore the function of EHHADH in OS, EHHADH siRNA was used to knock down the EHHADH expression in MG63 cells. The western blotting and qRT-PCR analysis indicated the knockdown efficiency (Figures 8(b) and 8(c)). Besides, to assess the role of EHHADH on the growth of the MG63 cells, a qRT-PCR assay was accomplished to detect the proliferation-related gene expression in the different treated groups. According to Figure 8(d), knockdown of the EHHADH expression markedly inhibit the proliferation rate of the MG63 cells than that of the NC siRNA group.

EHHADH, an L-bifunctional enzyme, is a part of the classical peroxisomal fatty acid *β*-oxidation pathway. A powerful way to trigger this pathway is the activation of the peroxisome proliferator-activated receptor *α* (PPAR*α*) [11]. The abnormal EHHADH expression can lead to several human diseases, such as Fanconi's syndrome and burn sepsis [12–14]. Previously, a high level of EHHADH has been found in various cancers, which can be correlated with cancer development, and therefore considered as a potential therapeutic target for cancers [15–18]. For instance, it was reported that EHHADH was a significant biomarker in renal cell carcinoma with a significant prognostic value [19–21]. Similarly, a recent study indicated that EHHADH was found to be correlated with the elucidation of the pathogenesis of hepatocellular carcinoma, and it was assumed that the EHHADH expression is an indicator of poor prognosis of hepatocellular carcinoma patients. However, the diagnostic and prognostic role of EHHADH in OS has not yet been fully understood.

RETRACTED

In the present research, we first sought to discover the clinical importance and prognostic value of EHHADH in OS patients with the help of clinical and the public database. Our results indicated that the EHHADH expression was upregulated in sarcoma tissues as compared to the normal tissues. Furthermore, compared with the adjacent bone tissues, human OS tissues showed the overexpression of EHHADH. Moreover, the statistical results revealed a clear relationship between the EHHADH expression and the survival of OS patients, which was further supported by multivariate and univariate analyses, indicating that EHHADH could be designed as a possible prognostic index to monitor the progress of OS.

Furthermore, to examine the influence of the expression of the EHHADH on the OS cell proliferation, the siRNA of EHHADH was developed and used to transfect the human MG63 cells. The qRT-PCR analysis was performed to measure the proliferation-related genes *Cyclin D1* and *Cyclin D3*, and the results indicated that the proliferation of OS cells can be repressed by knockout EHHADH in vitro. However, much more evaluation and validation should be performed to study the role of EHHADH in OS cells and investigate the underlying molecular mechanism of this correlation.

## 4. Conclusions

The research indicated that EHHADH possesses significant importance in the diagnosis and prognosis of OS, while the dismal prognosis of OS patients can be predicted by the expression level of EHHADH. Additionally, the inhibited proliferation of MG63 cells under the influence of the reduction of EHHADH also supported the conclusion that EHHADH may perform a function of a valuable prognostic biomarker for OS patients.

## Figures and Tables

**Figure 1:** Identification of differentially expressed genes in sarcoma base on the TCGA database. (a) The heat map of mRNA expression information of 263 sarcoma patients and 2 normal people. (b) The volcano result of included datasets.

**Figure 2:** GO and KEGG enrichment analysis results of differentially expressed genes. (a) The information of FDR and count of significantly enriched GO terms. (b) The information of category and count of significantly enriched GO terms. (c) The information of enrich factor, FDR, and count of enriched KEGG pathways.

RETRACTED

**Figure 3:** PPI network construction and hub genes identification of DEGs. (a) PPI network of DEGs constructed with Cytoscape. (b) DEGs in the network were ranked by degree. The top ten genes were EHHADH, ACOX1, AGXT, HMGCL, PIPOX, SLC27A2, DLD, ACADM, CAT, and DAO.

**Figure 4:** The prognostic values of hub genes in sarcoma. It is depicted that EHHADH was associated with shorter overall survival, and PIPOX, ACOX1, and SLC27A2 were associated with longer overall survival (*p* < 0.05).

**Figure 5:** The coexpressed genes of EHHADH in sarcoma ranked by correlation factor. The top ten genes were DMGDH, BHMT2, TMEM37, DAB2, TLR3, GAL3ST1, SLC5A10, SLC17A3, CHST13, and CID3B.

**Figure 6:** The prognostic values of coexpressed genes of EHHADH in sarcoma. DMGDH, BHMT2, TMEM37, TLR3, SLC17A3, and CID3B were associated with longer overall survival (*p* < 0.05).

**Figure 7:** GO and KEGG enrichment analysis results of EHHADH and its coexpressed genes. (a) Relationship and interactions between enriched GO terms. (b) Enriched KEGG pathways. hsa00983: drug metabolism-other enzymes, hsa00982: drug metabolism-cytochrome P450, hsa00980: metabolism of xenobiotics by cytochrome P450, hsa05204: chemical carcinogenesis, hsa01100: metabolic pathways, hsa00053: ascorbate and aldarate metabolism, hsa00040: pentose and glucuronate interconversions, hsa00860: porphyrin and chlorophyll metabolism, hsa00140: steroid hormone biosynthesis, hsa00830: retinol metabolism, and hsa00770: pantothenate and CoA biosynthesis. (c) Enriched GO terms. MF0001972: retinoic acid binding, MF0015020: glucuronosyltransferase activity, MF0016758: transferase activity, transferring hexosyl groups, CC0016324: apical plasma membrane, CC0070062: extracellular exosome, CC0005887: integral component of plasma membrane, BP1904224: negative regulation of glucuronosyltransferase activity, BP2001030: negative regulation of cellular glucuronidation, and BP0045922: negative regulation of fatty acid metabolic process.

**Figure 8:** Inhibition of EHHADH suppresses MG63 cell proliferation. (a) qRT-PCR results of the EHHADH expression in OS tissue and the bone tissue. (b) The level of EHHADH following the siRNA EHHADH treatment in MG63 cells. (c) qRT-PCR results of the EHHADH expression in MG63 cells receiving different treatments. (d) The expression of proliferation-related genes cyclin D1 and cyclin D3 in the different groups was assessed by qRT-PCR analysis. ^∗^*p* < 0.05, ^∗∗^*p* < 0.01, ^∗∗^*p* < 0.01. Data are the means ± SDs of three independent experiments.

RETRACTED

**Table 1:** GO function enrichment analysis of DEGs. Top 15 GO terms were selected.

Term	Name	Count	FDR
A, biological processes			
GO: 0008152	Metabolic process	46	1.50*E*-18
GO: 0007588	Excretion	20	5.97*E*-13
GO: 0006635	Fatty acid beta-oxidation	20	2.42*E*-11
GO: 0055085	Transmembrane transport	44	5.10*E*-11
GO: 0006814	Sodium ion transport	24	1.02*E*-09
GO: 0055114	Oxidation-reduction process	70	2.06*E*-09
B, molecular functions			
GO: 0009055	Electron carrier activity	25	5.06*E*-09
C, cellular components			
GO: 0070062	Extracellular exosome	317	1.51*E*-52
GO: 0016324	Apical plasma membrane	84	1.18*E*-39
GO: 0005759	Mitochondrial matrix	73	1.61*E*-26
GO: 0005739	Mitochondrion	147	1.97*E*-20
GO: 0031526	Brush border membrane	24	1.13*E*-15
GO: 0016323	Basolateral plasma membrane	41	8.68*E*-15
GO: 0005887	Integral component of plasma membrane	129	3.56*E*-11
GO: 0005782	Peroxisomal matrix	18	6.33*E*-10

**Table 2:** KEGG pathway enrichment analysis of DEGs. Top 20 KEGG pathways were selected.

KEGG pathways			
Term	Name	Count	FDR
hsa01100	Metabolic pathways	194	2.12*E*-41
hsa01130	Biosynthesis of antibiotics	53	5.46*E*-17
hsa00280	Valine, leucine, and isoleucine degradation	26	6.03*E*-17
hsa01200	Carbon metabolism	38	1.39*E*-16
hsa00630	Glyoxylate and dicarboxylate metabolism	17	7.89*E*-12
hsa00640	Propanoate metabolism	15	4.88*E*-09
hsa00071	Fatty acid degradation	17	3.06*E*-08
hsa04964	Proximal tubule bicarbonate reclamation	13	4.15*E*-08
hsa04146	Peroxisome	23	5.39*E*-08
hsa00620	Pyruvate metabolism	16	9.28*E*-08
hsa00020	Citrate cycle (TCA cycle)	14	1.13*E*-07
hsa00260	Glycine, serine, and threonine metabolism	15	4.71*E*-07
hsa00410	Beta-alanine metabolism	13	1.70*E*-06
hsa00650	Butanoate metabolism	12	2.90*E*-06
hsa00250	Alanine, aspartate, and glutamate metabolism	13	6.95*E*-06
hsa00380	Tryptophan metabolism	13	3.29*E*-05
hsa01212	Fatty acid metabolism	14	4.26*E*-05
hsa03320	PPAR signaling pathway	16	9.57*E*-05
hsa04966	Collecting duct acid secretion	10	1.95*E*-04
hsa00330	Arginine and proline metabolism	13	3.27*E*-04

**Table 3:** Functional and KEGG pathway enrichment analysis of EHHADH and its coexpressed genes. Top 3 GO terms and KEGG terms with *p* < 0.05 were selected.

Term	Name	Count	FDR
A, biological processes			
GO: 1904224	Negative regulation of glucuronosyltransferase activity	5	5.78*E*-07
GO: 2001030	Negative regulation of cellular glucuronidation	5	5.78*E*-07
GO: 0045922	Negative regulation of fatty acid metabolic process	5	5.78*E*-07
B, molecular functions			
GO: 0001972	Retinoic acid binding	5	8.33*E*-05
GO: 0015020	Glucuronosyltransferase activity	5	8.46*E*-05
GO: 0016758	Transferase activity, transferring hexosyl groups	5	8.46*E*-05
C, cellular components			
GO: 0016324	Apical plasma membrane	10	6.69*E*-06
GO: 0070062	Extracellular exosome	23	7.17*E*-05
GO: 0005887	Integral component of plasma membrane	13	9.71*E*-03
D, KEGG pathways			
hsa00983	Drug metabolism—other enzymes	7	4.20*E*-06
hsa00982	Drug metabolism—cytochrome P450	7	2.28*E*-05
hsa00980	Metabolism of xenobiotics by cytochrome P450	7	2.51*E*-05
hsa05204	Chemical carcinogenesis	7	2.51*E*-05
hsa01100	Metabolic pathways	19	2.51*E*-05
hsa00053	Ascorbate and aldarate metabolism	5	8.08*E*-05
hsa00040	Pentose and glucuronate interconversions	5	1.58*E*-04
hsa00860	Porphyrin and chlorophyll metabolism	5	3.67*E*-04
hsa00140	Steroid hormone biosynthesis	5	1.17*E*-03
hsa00830	Retinol metabolism	5	1.55*E*-03
hsa00770	Pantothenate and CoA biosynthesis	3	2.01*E*-02

RETRACTED

## Data Availability

The data used to support the findings of this study are available from the corresponding author upon request.

## References

[1] Chen R., Wang G., Zheng Y., Hua Y., Cai Z. (2019). Drug resistance-related microRNAs in osteosarcoma: translating basic evidence into therapeutic strategies. *Journal of Cellular and Molecular Medicine*.

[2] Roberts R. D., Lizardo M. M., Reed D. R. (2019). Provocative questions in osteosarcoma basic and translational biology: a report from the Children's oncology group. *Cancer*.

[3] Harrison D. J., Geller D. S., Gill J. D., Lewis V. O., Gorlick R. (2018). Current and future therapeutic approaches for osteosarcoma. *Expert Review of Anticancer Therapy*.

[4] Ouyang Z., Li H., Zhai Z. (2018). Zoledronic acid: pleiotropic anti-tumor mechanism and therapeutic outlook for osteosarcoma. *Current Drug Targets*.

[5] Rickel K., Fang F., Tao J. (2017). Molecular genetics of osteosarcoma. *Bone*.

[6] Wang Z., Wang Z., Li B., Wang S., Chen T., Ye Z. (2019). Innate immune cells: a potential and promising cell population for treating osteosarcoma. *Frontiers in Immunology*.

[7] He J., Zhao H., Deng D. (2020). Screening of significant biomarkers related with prognosis of liver cancer by lncRNA-associated ceRNAs analysis. *Journal of Cellular Physiology*.

[8] Peng H., Deng Y., Wang L. (2019). Identification of potential biomarkers with diagnostic value in pituitary adenomas using prediction analysis for microarrays method. *Journal of Molecular Neuroscience*.

[9] Vernia S., Cavanagh-Kyros J., Barrett T., Tournier C., Davis R. J. (2016). Fibroblast growth factor 21 mediates glycemic regulation by hepatic JNK. *Cell Reports*.

[10] Yeh C. S., Wang J. Y., Cheng T. L., Juan C. H., Wu C. H., Lin S. R. (2006). Fatty acid metabolism pathway play an important role in carcinogenesis of human colorectal cancers by microarray-bioinformatics analysis. *Cancer Letters*.

RETRACTED

[11] Houten S. M., Denis S., Argmann C. A. (2012). Peroxisomal L-bifunctional enzyme (Ehhadh) is essential for the production of medium-chain dicarboxylic acids. *Journal of Lipid Research*.

[12] Klootwijk E. D., Reichold M., Helip-Wooley A. (2014). Mistargeting of peroxisomal EHHADH and inherited renal Fanconi's syndrome. *The New England Journal of Medicine*.

[13] Xu X., Shi Z., Hu J. (2015). Identification of differentially expressed genes associated with burn sepsis using microarray. *International Journal of Molecular Medicine*.

[14] Marcus S. L., Miyata K. S., Zhang B., Subramani S., Rachubinski R. A., Capone J. P. (1993). Diverse peroxisome proliferator-activated receptors bind to the peroxisome proliferator-responsive elements of the rat hydratase/dehydrogenase and fatty acyl-CoA oxidase genes but differentially induce expression. *Proceedings of the National Academy of Sciences of the United States of America*.

[15] Duclos S., Bride J., Ramirez L. C., Bournot P. (1997). Peroxisome proliferation and beta-oxidation in Fao and MH1C1 rat hepatoma cells, HepG2 human hepatoblastoma cells and cultured human hepatocytes: effect of ciprofibrate. *European Journal of Cell Biology*.

[16] Xiao H., Chen P., Zeng G. (2019). Three novel hub genes and their clinical significance in clear cell renal cell carcinoma. *Journal of Cancer*.

[17] Gao X., Wang X., Zhang S. (2018). Bioinformatics identification of crucial genes and pathways associated with hepatocellular carcinoma. *Bioscience Reports*.

[18] Suto K., Kajihara-Kano H., Yokoyama Y. (1999). Decreased expression of the peroxisomal bifunctional enzyme and carbonyl reductase in human hepatocellular carcinomas. *Journal of Cancer Research and Clinical Oncology*.

[19] Litwin J. A., Beier K., Völkl A., Hofmann W. J., Fahimi H. D. (1999). Immunocytochemical investigation of catalase and peroxisomal lipid beta-oxidation enzymes in human hepatocellular tumors and liver cirrhosis. *Virchows Archiv*.

[20] Meyer K., Jia Y., Cao W. Q., Kashireddy P., Rao M. S. (2002). Expression of peroxisome proliferator-activated receptor alpha, and PPARalpha regulated genes in spontaneously developed hepatocellular carcinomas in fatty acyl-CoA oxidase null mice. *International Journal of Oncology*.

[21] Wen Q., Wang D., Yang Y. (2017). Competing endogenous RNA screening based on long noncoding RNA-messenger RNA co-expression profile in hepatitis B virus-associated hepatocarcinogenesis. *Journal of Traditional Chinese Medicine*.

